# An IoT-Based Motion Tracking System for Next-Generation Foot-Related Sports Training and Talent Selection

**DOI:** 10.1155/2021/9958256

**Published:** 2021-06-25

**Authors:** Shanshan Lu, Xiao Zhang, Jiangqing Wang, Yufan Wang, Mengjiao Fan, Yu Zhou

**Affiliations:** ^1^Department of Computer Science, South-Central University for Nationalities, Wuhan 430074, China; ^2^Department of Industrial Engineering & Management, School of Mechanical Engineering, Shanghai Jiao Tong University, Shanghai 200240, China; ^3^College of Computer Science and Software Engineering, Shenzhen University, Shenzhen, China

## Abstract

Motion tracking in different fields (medical, military, film, etc.) based on microelectromechanical systems (MEMS) sensing technology has been attracted by world's leading researchers and engineers in recent years; however, there is still a lack of research covering the sports field. In this study, we propose a new AIoT (AI + IoT) paradigm for next-generation foot-driven sports (soccer, football, takraw, etc.) training and talent selection. The system built is cost-effective and easy-to-use and requires much fewer computational resources than traditional video-based analysis on monitoring motions of players during training. The system built includes a customized wireless wearable sensing device (WWSDs), a mobile application, and a data processing interface-based cloud with an ankle attitude angle analysis model. Eleven right-foot male participators wore the WWSD on their ankle while each performed 20 instances of different actions in a formal soccer field. The experimental outcome demonstrates the proposed motion tracking system based on AIoT and MEMS sensing technologies capable of recognizing different motions and assessing the players' skills. The talent selection function can partition the elite and amateur players at an accuracy of 93%. This intelligent system can be an emerging technology based on wearable sensors and attain the experience-driven to data-driven transition in the field of sports training and talent selection and can be easily extended to analyze other foot-related sports motions (e.g., taekwondo, tumble, and gymnastics) and skill levels.

## 1. Introduction

Recent trends in smart wearable technologies based on the Internet of Things (IoT) have opened up a large number of applications [1], which involve the recognition of sports activities [2–4]. Soccer, also known as football in some countries, is one of the most popular sports in the world with numerous professionals and an even larger number of nonprofessional practitioners. Soccer players train a specific set of well-defined motions (e.g., shooting and passing) to consolidate them into muscle memory and lower their reaction time during a game. The correct execution of the exercises and training has a steep learning curve. Quantity and quality information about soccer motions like shooting and passing an exhaustive performance evaluation is indispensable for coaches and players in training sessions and competitions.

Traditionally, the training of professional soccer players is human-oriented, which is done by subjective guidance based on the personal experience of coaching staff or trainers. However, different coaches could have different ideas upon their experience, and there are many fast and slight soccer motions during an action that cannot be captured through their visual sense. The need for an objectively and digitized method rather than a subjective method is raised. In the last few years, there have appeared lots of research efforts in the field of professional soccer for a measurable and quantifiable analysis of sports through information technology. The manager and coaching staff use videography to monitor the biomechanics of soccer actions and check the objective players' performance [5]. Despite this, videography is typically restricted by equipment and environment and unable to give feedback to the coaching staff or soccer players in real time due to the significant amounts of storage and computational load.

The rapid development of bluetooth low energy (BTLE) and microelectromechanical systems (MEMS) technologies implements durative motion data capture and communication in real time. There is increasing research on motion recognition by using inertial low-cost sensors worn on the body. For example, the authors of [3] use inertial sensors worn on the wrist to identify the stroke type of table tennis. In [6, 7], wearable sensing devices (WSDs) on the wrist are used to classify different volleyball and badminton actions. However, due to the nature of soccer, the ankle movements of players are complex and indicative of different soccer motions. Moreover, the high variability in the training and individual execution of each exercise makes the classification of soccer motions extremely challenging. A particular challenge we address is to classify the most fundamental soccer motions (i.e., shooting and passing) (the development process and methods we describe in this paper can be reused in more motion recognition applications). The existing approaches used in other sports are hardly applicable [8].

Therefore, an IoT system based on WSD is proposed in this work to provide objective feedback to coaches and soccer players after or during a training session to help them improve their skills. The proposed IoT system consists of wearable devices, a mobile device (e.g., a mobile phone or tablet), and a data processing platform based cloud. A WSD of MEMS is used to collect raw data from soccer players. By using BTLE technology, the material is transmitted to the cloud-based data processing platform, which analyzes the data and outputs the results to a mobile device in real time. A support vector machine (SVM) model classification algorithm with an ankle-based attitude angle model is proposed to recognize different motions and assess different skill levels.

This system is ideally suitable for the young player soccer training. A soccer training session typically includes exercises of passes, crosses, and shots For example, in a soccer club or training school, there are dozens or hundreds of young players conducting an exercise of shooting or passing. It is evident that a limited number of coaches are hard to assess all soccer players' individual execution of each exercise. Instead, by using our developed system, how many passes/shoots have been done and how professional will be shown on a coach's mobile device. The work we present enables soccer players to keep track of the training exercises they perform. The managers and coaches could get an overview of the exercises during past days, weeks, or months, which they could use to arrange future training sessions pointedly. We intend to apply the system in a realistic training environment with a focus on the recognition of basic soccer motions. This study demonstrates the trend in using the IoT framework for a new era of soccer training.

Our key novelty and main contributions are summarized as follows:

- We develop an IoT system for soccer motion recognition and assessment, in which a WSD with overall dimensions of 2 mm × 10.3 mm × 8.7 mm is developed to capture inertial data; a mobile application allows visualization of experimental outputs and transfers the data to the cloud-based processing platform.
- We build a SVM classification algorithm with an attitude angle model to classify different soccer motions and make a distinction between the skill levels between elite and amateur players.
- Our system is confirmed by the experimental results that it enables recognizing different motions, that is, shooting and passing, with an accuracy close to 90%. The talent selection distinguishes between the elite and amateur players with an accuracy of 93%.

We organize the remainder main structure of this article as follows: we give a literature review in Section 2. Then, we illustrate the system composition and data acquisition in Section 3. Next, Section 4 presents our algorithm for soccer motion recognition and assessment as well as the experimental results. Finally, Section 5 summarizes the contribution.

## 2. Related Work

Motion analysis and recognition by using information technology have been a field of study for decades. During this period, a variety of motion recognition applications and approaches have been proposed to assess the performance and correctness of a physical exercise of an athlete and provide feedback to users about their actions.

In early studies, motion recognition was a kind of computer vision field that recognizes human pose or action, in which video image acquisition and processing technology was adopted to identify the human body's motion behavior. In vision-based action recognition, the training method is mainly to collect videos, images, and other information to analyze the moving process. Therefore, it is necessary to place cameras and other monitors in advance in the detection environment for data collection. The popularity of the RGB camera has made it an effective auxiliary tool for the human motion recognition study and also leads to the appearance of several survey articles [9, 10] discussing various features and classifiers for human action recognition. Though image analysis technology can identify people's daily moves more accurately, image analysis technology still suffers from many shortcomings. In nature, a large number of hardware conditions are required so as to run computer vision algorithms and computationally concentrated image processing. Moreover, a large amount of image data acquired suffers from insufficient storage, leading to failure in monitoring [11].

Several human activities' recognition approaches have been presented, in which wearable sensors with accelerometers and gyroscopes are used to acquire motion data [12, 13]. A much wider field of views can be obtained by this sensor technology. Long-running recordings, calculation, and constant interaction are possible owing to the progress of inertial sensors in energy-consuming reduction and the improvement of computational power. Moreover, 3D motion data which consists of 3-axis angular velocities from gyroscopes as well as 3-axis accelerations from accelerometers can be given by wearable inertial sensors [14, 15].

Sensors are often of small size, high precision and sensitivity, and low environmental requirements and power consumption, as well as easy to wear. A universal activity recognition depth framework based on multimodal wearable sensors was proposed in [16, 17]. Shoaib et al. [18] used inertial sensors to detect the activities that involve hand gestures (smoking, eating, drinking, giving a chat, etc.). In the field of competitive sports, most movement recognition systems are dedicated to solving wrist movements or simple lower limb movements such as walking and standing [19].

There are a few studies on the recognition and assessment of soccer players' motions. Reference [20] indicated that soccer players' shin guards instrumented with sensors can measure ankle joint kinematics. Meamarbashi et al. tested whether sensors can be used to examine kinematic parameters of soccer players in [21], but no further analysis of the data. In [4], Haladjian et al. developed a smart glove with an inertial sensor and gave a machine learning algorithm to recognize the goalkeeper's training exercises, which was a good attempt to use WSD to recognize soccer motion. As far as we know, this is the first work to use a single WSD attached to an ankle to recognize different soccer players' motions (not just the goalkeepers) and assess their skill levels.

## 3. System Design and Data Acquisition

Though WSDs have been widely used in motion recognition, for soccer motions, the existing approaches are hardly applicable. However, the limited number of coaches are hard to assess all soccer players' individual performance. Thus, this study presents a complete system in using the IoT framework for soccer motion recognition. By using the developed system, the passes/shoots and their skill levels can be shown on a mobile device hold by a coach. The system enables soccer players to keep track of the training exercises they perform. The specific details of hardware design, interface software, and data acquisition are given in this section.  Figure 1 shows an overview of our IoT system for soccer motion recognition and assessment, which is composed of wireless WSDs, mobile devices, and cloud-based data processing platform.

By using the proposed IoT system, BTLE sent mobile device data collected by WSD. It transfers the raw data to the remote execution server via cloud computing technology at the moment when the mobile device received the exercise data. Completing all data collection and processing, users can view the analysis results of soccer players through the platform.

### 3.1. Hardware and Software System

We collect data using a wireless WSD, jointly developed by our team and the company *AI Motion Sports* (https://www.aimotionsports.com/en/).  Figure 2 shows the components of the device. This wireless WSD is comprised of four major components: an MEMS motion sensing chip with a 3-axis gyroscope and accelerometer, a microprocessing unit with Bluetooth wireless newsletter function, a lithium battery, and an ON-OFF switch on the back of the board.

The 3-axis gyroscope and accelerometer in MEMS are used to sense the motions and transform the signal into raw data. DA14583 Programmed in Dialog Semiconductor, Reading, UK, baseband radio processor and entirely integrates radio transceiver for BTLE. Not only is the microprocessor with chip nRF52832 characterized by low energy consumption but also highly efficient transmission by using Bluetooth v5.0. BMI160 from BOSCH has a fitting sensor range and tiny size (2.5 mm × 3.0 mm × 0.83 mm) [22] to enable it to be adopted.

The acceleration and orientation in three dimensions can be obtained through the high-integration and low-power BMI160. The entire WSD keep in size within 10.3 mm × 8.7 mm × 2 mm, using this IMU chip, weighing only 2 g. We develop a mobile application for receiving and visualizing data transmitted from WSD in real time. The application developed by the Java Script consists of three functional modules: wireless connection, real-time captured data demonstration, and data synchronization to the cloud. All data sensed are display synchronously and saved locally. A cloud-based approach is also used to save data received to a remote server. Once the data collection process is completed, user clients can access the analytical results.

### 3.2. Data Collection

We conduct the experiments at the Chinese Football Association (CFA) Youth Academy (Wuhan) (Chinese National Football Team Training Center) and Sports Center of South-Central University for Nationalities. We recruited 11 male soccer players, including 5 elites and 6 amateurs who are right-footed players. Among them, elite players had represented their club as participants in more than ten 10 national games from CFA Youth Academy (Wuhan); amateurs were beginners from university. As soccer is a foot-based sport, our small and light WSD is attached to each right-footed subject' right ankle when performing soccer basic training to make sure that major inertial data of soccer motions can be captured without obstruction. During the experiment, each subject performed 20 passings with the inside of the foot and 20 shootings with foot-arch at the soccer field of CFA Youth Academy (Wuhan). The subject performed the actions at the same position. Each subject's passings and shootings are required to be performed within a certain range of speed and precision; otherwise, we considered it was an invalid action and we did not count it.  Figure 3 illustrates our experimental scene.

Figure 4 displays the six-axis synchronal raw data captured by the WSD from elites by performing different soccer motions. The angular velocity as well as acceleration for passing are displayed in Figures 4(a) and 4(b), while Figures 4(c) and 4(d) show the related data information for shooting.

## 4. Soccer Motion Recognition and Assessment

The process of the soccer motion recognition system, as shown in Figure 5, can be divided into five steps: data preprocessing, attitude angle modeling, feature extraction and selection, dimensionality reduction, and classification. To be specific, the ankle-based attitude angles' features act a pivotal part in improving the accuracy of classification, since soccer as a type of foot-based sport is more complicated than other sports like racket sports. Principle component analysis (PCA) is adopted in our system to balance the complexity and the accuracy. Finally, we propose a SVM-based classification algorithm to recognize the soccer motions.

In data preprocessing, a 3-point moving average filter is used to lessen the noisy interference from raw data. By locating the peak of the signal, the segmentation of the motion signal can be processed automatically. The sliding-window algorithm [23] can be applied to process the signals in real time.

### 4.1. Angle Trajectory Model

As shown in Figure 6, the intuitive signal of {*ω*_*x*_, *ω*_*y*_, *ω*_*z*_} (acceleration from three dimensions: *x* -axis, *y* -axis, and *z* -axis) and {*α*_*x*_, *α*_*y*_, *α*_*z*_} (angular velocity from three dimensions) are not significant. We present an attitude angle model for extracting more useful features.

For sports motion recognition, angular velocity and acceleration are important features. Besides, the ankles' rotations are specially important for soccer motion recognition and assessment [16]. A three-dimensional rotation problem is typically addressed by a rotation matrix. Mining the information of attitude angle can improve characterizing the action. The attitude angle is expressed by three Euler angles: yaw, pitch, and roll.  Figure 7 shows the specific transformation.

The quaternion [24] as the quotient of two directed lines in a three-dimensional space is used to solve angle in the angle trajectory model. The representation of the quaternion is *p*=*p*_*ω*_+*p*_*x*_*i*+*p*_*y*_*j*+*p*_*z*_*k* with a real part *p*_*ω*_ and three imaginary parts parameters *p*_*x*_, *p*_*y*_, and *p*_*z*_. Calculate the initial attitude angle:

(1) $$\begin{array}{c} \left\{\begin{array}{c} \theta =\text{arcsin}\left(a_{x0}\right),\\ \varphi =\text{arctan}\frac{magy_{0}}{magx_{0}},\\ \psi =\text{arctan}\left(-\frac{a_{y0}}{a_{z0}}\right), \end{array}\right) \end{array}$$

where *a*_*x*0_, *a*_*y*0_, *a*_*z*0_ represent the initial acceleration; *θ*, *ψ*, and *φ* represent the initial yaw, roll, and pitch, respectively. mag*x*_0_ and mag*y*_0_ are calculated by *a*_*x*0_, *a*_*y*0_, *a*_*z*0_, specifically, mag*x*_0_ = *a*_*x*0_*a*_*y*0_+*a*_*x*0_*a*_*z*0_/1 − 2(*a*_*y*0_^2^+*a*_*z*0_^2^), and mag*y*_0_ = *a*_*x*0_*a*_*y*0_+*a*_*y*0_*a*_*z*0_/1 − 2(*a*_*x*0_^2^+*a*_*z*0_^2^) [25]. The initial four elements are calculated from the initial angle:

(2) $$\begin{array}{c} \left[\begin{array}{c} p_{0}\\ p_{1}\\ p_{2}\\ p_{3} \end{array}\right]=\left[\begin{array}{c} \sin\frac{\psi }{2}\sin\frac{\theta }{2}\sin\frac{\varphi }{2}+\cos\frac{\psi }{2}\cos\frac{\theta }{2}\cos\frac{\varphi }{2}\\ \sin\frac{\psi }{2}\cos\frac{\theta }{2}\cos\frac{\varphi }{2}-\cos\frac{\psi }{2}\sin\frac{\theta }{2}\sin\frac{\varphi }{2}\\ \cos\frac{\psi }{2}\sin\frac{\theta }{2}\cos\frac{\varphi }{2}+\sin\frac{\psi }{2}\cos\frac{\theta }{2}\sin\frac{\varphi }{2}\\ \cos\frac{\psi }{2}\cos\frac{\theta }{2}\sin\frac{\varphi }{2}-\sin\frac{\psi }{2}\sin\frac{\theta }{2}\cos\frac{\varphi }{2} \end{array}\right]. \end{array}$$

The Runge–Kutta method [26] which mainly eliminates the complicated process of solving differential equations when the derivatives and initial value information of the equation are known is used to solve four elements:

(3) $$\begin{array}{c} {\left[\begin{array}{c} p_{0}\\ p_{1}\\ p_{2}\\ p_{3} \end{array}\right]}_{t+△t}={\left[\begin{array}{c} p_{0}\\ p_{1}\\ p_{2}\\ p_{3} \end{array}\right]}_{t}+\frac{△t}{2}\left[\begin{array}{c} -\omega_{x}\cdot p_{1}-\omega_{y}\cdot p_{2}-\omega_{z}\cdot p_{3}\\ +\omega_{x}\cdot p_{0}-\omega_{z}\cdot p_{2}-\omega_{y}\cdot p_{3}\\ +\omega_{y}\cdot p_{0}-\omega_{z}\cdot p_{1}+\omega_{x}\cdot p_{3}\\ -\omega_{z}\cdot p_{0}+\omega_{y}\cdot p_{1}-\omega_{x}\cdot p_{2} \end{array}\right], \end{array}$$

where *t* means the current time value and △*t* represents the interval of next data. The following uses the quaternion to solve the attitude angle. The coordinate transformation matrix *D* of the known object coordinate system to the Earth coordinate system is

(4) $$\begin{array}{c} D=\left[\begin{array}{ccc} 1 & 0 & 0\\ 0 & 1 & 0\\ 0 & 0 & 1 \end{array}\right]+2\;\cos\frac{\theta }{2}\left[\begin{array}{ccc} 0 & -n\;\sin\frac{\theta }{2} & m\;\sin\frac{\theta }{2}\\ n\;\sin\frac{\theta }{2} & 0 & -l\;\sin\frac{\theta }{2}\\ -m\;\sin\frac{\theta }{2} & l\;\sin\frac{\theta }{2} & 0 \end{array}\right]\\ +2\left[\begin{array}{ccc} -\left(m^{2}+n^{2}\right)\sin^{2}\frac{\theta }{2} & lm\;\sin^{2}\frac{\theta }{2} & nl\;\sin^{2}\frac{\theta }{2}\\ lm\;\sin^{2}\frac{\theta }{2} & -\left(l^{2}+n^{2}\right)\sin^{2}\frac{\theta }{2} & mn\;\sin^{2}\frac{\theta }{2}\\ nl\;\sin^{2}\frac{\theta }{2} & mn\;\sin^{2}\frac{\theta }{2} & -\left(m^{2}+l^{2}\right)\sin^{2}\frac{\theta }{2} \end{array}\right]. \end{array}$$

*m*, *l*, and *n* mean the direction vector projected onto the geographic coordinate along the direction of rotation vector. The rotation of the object corresponds to the rotation around the axis. The trigonometry of a quaternion is $\cos\theta /2+\left(l\overset{⟶}{i}+m\overset{⟶}{j}+n\overset{⟶}{k}\right)\sin\theta /2=\cos\theta /2+\overset{⟶}{u}\sin\theta /2$, in which $\overset{⟶}{i},\overset{⟶}{j},\overset{⟶}{k}$ denote the unit direction vector in the geographic graticule system:

(5) $$\begin{array}{c} \left\{\begin{array}{c} p_{0}=\cos\frac{\theta }{2},\\ p_{1}=l\;\sin\frac{\theta }{2},\\ p_{2}=m\;\sin\frac{\theta }{2},\\ p_{3}=n\;\sin\frac{\theta }{2}. \end{array}\right) \end{array}$$

The constructed quaternion describes the fixed-point rotation problem of the substance. Correspondingly, the object system is formed by one-time equivalent rotation of the Earth system. Equation (5) is substituted into *D*_1_:

(6) $$\begin{array}{c} D_{1}=\left[\begin{array}{ccc} p_{0}^{2}+p_{1}^{2}-p_{2}^{2}-p_{3}^{2} & 2\left(p_{1}p_{2}-p_{0}p_{3}\right) & 2\left(p_{0}p_{2}+p_{1}p_{3}\right)\\ 2\left(p_{0}p_{3}+p_{1}p_{2}\right) & p_{0}^{2}-p_{1}^{2}+p_{2}^{2}-p_{3}^{2} & 2\left(p_{2}p_{3}-p_{0}p_{1}\right)\\ 2\left(p_{1}p_{3}-p_{0}p_{2}\right) & 2\left(p_{0}p_{1}+p_{2}p_{3}\right) & p_{0}^{2}-p_{1}^{2}-p_{2}^{2}+p_{3}^{2} \end{array}\right]. \end{array}$$

Let the unit vector in the coordinate system *X* be (*ex*_1_, *ey*_1_, *ez*_1_)^*T*^ and correspond to (*ex*_2_, *ey*_2_, *ez*_2_)^*T*^ in *Y*, and the direction of the projection of the (*ex*_2_, *ey*_2_, *ez*_2_)^*T*^ is *C*_*b*_^*n*^. Suppose there is a vector *R* whose magnitude on *X* is (*x*, *y*, *z*)^*T*^ and on *Y* is (*x*_2_, *y*_2_, *z*_2_)^*T*^; then, coordinate transformation is (*x*, *y*, *z*)^*T*^=*C*_*b*_^*n*^(*x*_2_, *y*_2_, *z*_2_)^*T*^. The attitude angle transformation matrix is also converted into the coordinate transformation matrix form of object coordinate system to a geographic coordinate system and *C*_*b*_^*n*^ is obtained as follows:

(7) $$\begin{array}{c} C_{b}^{n}=Rot\left(z,\psi \right)Rot\left(y,\theta \right)Rot\left(x,\varphi \right)\\ =\left[\begin{array}{ccc} \cos\;\psi & -\sin\;\psi & 0\\ \cos\;\psi & \cos\;\psi & 0\\ 0 & 0 & 1 \end{array}\right]\left[\begin{array}{ccc} 1 & 0 & 0\\ 0 & \cos\;\varphi & -\sin\;\varphi \\ 0 & \sin\;\varphi & \cos\;\varphi \end{array}\right]\left[\begin{array}{ccc} \cos\;\theta & 0 & \sin\;\theta \\ 0 & 1 & 0\\ -\sin\;\theta & 0 & \cos\;\theta \end{array}\right]\\ =\left[\begin{array}{ccc} \cos\;\psi \;\cos\;\theta & -\sin\;\psi \;\cos\;\varphi +\cos\;\psi \;\sin\;\theta \;\sin\;\varphi & \sin\;\psi \;\sin\;\varphi +\cos\;\psi \;\sin\;\theta \;\cos\;\varphi \\ \sin\;\psi \;\cos\;\theta & \cos\;\psi \;\cos\;\varphi +\sin\;\psi \;\sin\;\theta \;\sin\;\varphi & -\cos\;\psi \;\sin\;\varphi +\sin\;\psi \;\sin\;\theta \;\cos\;\varphi \\ -\sin\;\theta & \cos\;\theta \;\sin\;\varphi & \cos\;\theta \;\cos\;\varphi \end{array}\right]. \end{array}$$

Both *D*_1_ and *C*_*b*_^*n*^ are matrices transforming the object coordinate system attitude into the geographic coordinate system; that is,

(8) $$\begin{array}{c} \left\{\begin{array}{c} 2\left(p_{1}p_{3}-p_{0}p_{2}\right)=-\sin\;\theta =g_{1},\\ 2\left(p_{0}p_{1}+p_{2}p_{3}\right)=\sin\;\varphi \;\cos\;\theta =g_{2}m,\\ p_{0}^{2}-p_{1}^{2}-p_{2}^{2}+p_{3}^{2}=\cos\;\theta \;\cos\;\varphi =g_{3},\\ 2\left(p_{0}p_{3}+p_{1}p_{2}\right)=\sin\;\psi \;\cos\;\theta =g_{4},\\ p_{0}^{2}+p_{1}^{2}-p_{2}^{2}-p_{3}^{2}=\cos\;\psi \;\cos\;\theta =g_{5}. \end{array}\right) \end{array}$$

The equation for solving the attitude angle by the quaternion is

(9) $$\begin{array}{c} \left\{\begin{array}{c} \text{roll}=\text{arctan}\frac{2\left(p_{0}p_{3}+p_{1}p_{2}\right)}{1-2\left(p_{0}^{2}+p_{1}^{2}\right)},\\ \text{pitch}=\text{arctan}\frac{2\left(p_{1}p_{3}-p_{0}p_{2}\right)}{4{\left(p_{0}p_{3}+p_{1}p_{2}\right)}^{2}+{\left(1-2\left(p_{0}^{2}+p_{1}^{2}\right)\right)}^{2}},\\ \text{yaw}=\text{arctan}\frac{2\left(p_{0}p_{1}+p_{2}p_{3}\right)}{1-2\left(p_{2}^{2}+p_{3}^{2}\right)}. \end{array}\right) \end{array}$$

The frequency of the sensor repetition rate is 100Hz. Then, the angular velocity value is substituted into the solution attitude angle *A*_*n*−*i*_.  Figure 8 shows the comparison of attitude angle of elites and amateurs.

By combining *A*_*n*−*i*_ with *S*_*n*−*i*_ as a part of *R*_*n*−*i*_, we extract the basic and morphology features *f*_*ni*_ of segments *R*(*n*)_*i*_, as shown in Table 1.

*F*(*n*)=(*f*_1_,…, *f*_*mn*_) are merged into one large matrix *F* of size *n* × *m*. The updated data form is shown in Figure 9.

### 4.2. Principle Component Analysis

The cloud server benefits from reducing memory requirements, computing load, and necessary bandwidth during model implementation. To represent identified variables in compact feature variables, we perform PCA processing. The model with PCA can achieve higher accuracy than other nonlinear dimensionality reduction methods [7]. PCA is essentially a base transformation that makes transformed data have the largest variance, which means the variance between one axis (spindle) and the point is minimized by the rotation of the coordinate axis and the translation of the coordinate origin. Suppose the matrix *F* with the dimension of *n* × *m*, which means that there is total *n* samples in *m*-dimensions. *F* can be decomposed into *U*Σ*V*^*T*^, where *U* has the same size as *F*, and the orthogonal matrix *V* is *m* × *m*, Σ is a diagonal matrix of the same size as *V*. Then, *Y*_*r*_*U*Σ_*r*_=*F*(Σ*V*^*T*^)^(−1)^Σ_*r*_.

We extracted a total of 34-dimensional features for a vector characterizing, where *F*=[*F*_1_, *F*_2_,…, *F*_34_]. After PCA, the obtained new features can be expressed as *Y*_*r*_=[*Y*_*r*1_, *Y*_*r*2_,…, *Y*_*rm*_] and *m* represents the calculated dimension:

(10) $$\begin{array}{c} Y_{rm}=F_{1}a_{ij}+F_{2}a_{ij}+\cdots +F_{m}a_{ij}, \end{array}$$

where *a*_*ij*_ are eigenvalues of the covariance matrix. Equation (10) can be simplified as follows:

(11) $$\begin{array}{c} Y_{rm}=F_{1}a_{1}+F_{2}a_{2}+\cdots +F_{m}a_{m}. \end{array}$$

### 4.3. Support Vector Machine

SVM is widely applied in the domain of machine learning and pattern recognition as a tool to solve the classification problem. The basic model of SVM aims to maximize the distance of the closet samples which is called support vector to the hyperplane on the eigenspace [27]. In SVM, a training data point is regarded as a $p$-dimensional vector; the objective is to separate such points using a $(p-1)$-dimensional hyperplane [19]. That is, the training points are mapped to points in space to maximize the width of the gap between the two and several categories by SVM. Compared to other supervised algorithms such as logistics regression (LR) model or Naïve Bayes algorithm [28], the SVM algorithm is more suitable to deal with high-dimensional and linear inseparable problems by freely selecting the parametric model and only use support vector as the classification basis of hyperplane which meets our expectations as our problem is a small sample linear inseparable problem.

The training dataset is set as *T*={(*X*_*k*_, *y*_*k*_)*|X* ∈ *R*^*m*^, *y*_*k*_ ∈ {0,1}_*k*=1_^*n*^}. Here are total *n* samples. *X* represents an *m*-dimensional matrix, the value of the classification label *y*_*k*_ is 0 or 1, and the current sample is *X*_*k*_. Therefore, the representation of the optimization objective function is

(12) $$\begin{array}{c} \underset{\omega ,b}{\min}\frac{1}{2}{\left\|\omega \right\|}^{2},\\ \begin{array}{cc} \mathrm{s.t}\text{.} & y_{k}\left(\omega \cdot x_{k}+b\right)-1\geq 0,k=1,2,\ldots ,N \end{array}. \end{array}$$

Here, *ω* is a vector on a hyperplane and the offset *b* of the superflat is along *ω* from the origin. Problem (12) is a convex quadratic programming problem [29]. According to the convex optimization theory, transform problem (12) into an unconstrained problem. The optimization function can be denoted as

(13) $$\begin{array}{c} L\left(\omega ,b,\alpha \right)=\frac{1}{2}{\left\|\omega \right\|}^{2}-\sum_{k=1}^{N}\alpha_{k}y_{k}\left(\omega \cdot x_{k}+b\right)+\sum_{k=1}^{N}\alpha_{k}, \end{array}$$

where *α*_*k*_ is a Lagrangian multiplier, *α*_*k*_ ≥ 0, (*k*=1,2,3,…, *n*). The original problem is expressed as

(14) $$\begin{array}{c} \underset{\alpha }{\max}\underset{\omega b}{\min}L\left(\omega ,b,\alpha \right). \end{array}$$

*α*_*k*_ is a Lagrangian multiplier where *α*_*k*_ ≥ 0, (*k*=1,2,3,…, *n*). Solving *ω* and *b* as a minimum problem, we can get the value of *ω* and *b*:

(15) $$\begin{array}{c} \left\{\begin{array}{c} \omega =\sum_{k=1}^{N}\alpha_{k}y_{k}x_{k},\\ \sum_{k=1}^{N}\alpha_{k}y_{k}=0. \end{array}\right) \end{array}$$

Substituting the obtained solution into the Lagrangian function for a minimize problem, the following optimization function can be obtained after substituting:

(16) $$\begin{array}{c} s\mathrm{.t}\text{.}\begin{array}{c} \underset{\alpha }{\min}\frac{1}{2}\sum_{k=1}^{N}\sum_{j=1}^{N}\alpha_{i}\alpha_{j}y_{k}y_{j}\left(x_{k}\cdot x_{j}\right)-\sum_{k=1}^{N}\alpha_{k}\\ \sum_{k=1}^{N}\alpha_{k}y_{k}=0\\ \alpha_{k}\geq 0,k=1,2,\ldots ,N. \end{array} \end{array}$$

Then, introduce a slack variable *ζ*_*k*_ for (*x*_*k*_, *y*_*k*_) for some abnormal sample points make the training set linearly inseparable. The penalty parameter *C* ≥ 0. The original issue is described as

(17) $$\begin{array}{c} \mathrm{s.t}\text{.}\begin{array}{c} \underset{\omega ,b,\zeta }{\min}\frac{1}{2}{\left\|\omega \right\|}^{2}+C\sum_{k=1}^{N}\zeta_{k}\\ y_{k}\left(\omega \cdot x_{k}+b\right)\geq 1-\zeta_{k},k=1,2,\ldots ,N\\ \zeta_{k}\geq 0,k=1,2,\ldots ,N. \end{array} \end{array}$$

The ultimate function is obtained after conversion:

(18) $$\begin{array}{c} \mathrm{s.t}\text{.}\begin{array}{c} \underset{\alpha }{\min}\frac{1}{2}\sum_{k=1}^{N}\sum_{j=1}^{N}\alpha_{k}\alpha_{j}y_{k}y_{j}\left(x_{k}\cdot x_{j}\right)-\sum_{k=1}^{N}\alpha_{k}\\ \sum_{k=1}^{N}\alpha_{k}y_{k}=0\\ 0\leq \alpha_{k}\leq C,k=1,2,\ldots ,N. \end{array} \end{array}$$

There are two labels: passing and shooting represented by 0 and 1, respectively, in the action classification experiment. We obtained 264 sets for passing and 250 sets for shooting. The datasets are randomly divided into training and test sets, 80% of them used for training and the rest used as test data. Randomly selected parameters are shown in Table 2. The selectable parameter *C* ranges from 1 to 50000; *γ* range is from 0.00001 to 0.05, and the kernel function includes Linear, RBF, Sigmoid, and Polynomial. In order to solve overfitting, 3-fold cross is adopted. Experimental results show that *C*=1, *γ* is 0.0001, and linear kernel function is used in the optimal model.

We use the proposed SVM-based classifier to recognize the shooting and passing. Decision Tree [30] and K-nearest neighbor algorithm (KNN) [31] are the competitors in our experiments. The accuracy of different models for soccer motion recognition can be found in Table 3. Apparently, our proposed SVM-based algorithm has better performance than other competitors. The one with the attitude angle has a better performance than the others.

Table 4 shows the recognition and assessment results of our proposed system. The recognition accuracies for passing and shooting are 85.7% and 88.5% which illustrated a clear distinction between passing and shooting. The accuracy of classifying different behaviors can be 87.1% on average. This result suggests our system works.

### 4.4. Talent Selection System

Similar to the above analysis, the labels are elites and amateurs in the talent selection experiment. The selectable parameters are still randomly selected from Table 2. Thre-fold cross-validation is used again to prevent overfitting. Finally, the best performing classifiers are selected. Experimental results show that *C*=1 and linear kernel function applies to all optimal models. As for *γ*, different from motion recognition, the value is 0.00005.

As shown in Table 5, the accuracies of shooting level classifiers are higher than others. There is a clear difference between different level participants when shooting. The results show that the SVM with the attitude angle model also has satisfactory accuracy.

The results in Table 6 are all inferior to others, which means there might be little difference between participants when passing. As listed in Tables 3, 5, and 6, comparing with KNN and Decision Tree, SVM demonstrated superiority in dealing with the linear inseparable problem, and the one with attitude angle is better than the other.

As shown in Table 7, the assessment results of proposed system. Our model with attitude angle features obviously performs better than typical model. The professionals and amateurs are 88.7% and 85.1%, respectively, for passing. For the shooting action, the accuracy of the model is 93%, which also signifies that, for the shooting action, the skill gap between the professional and the amateur is bigger than the passing action.

## 5. Conclusion and Discussion

An AIoT system to recognize different soccer (football) motions and assess the skill levels of soccer players was proposed in this paper. The proposed IoT system consists of wearable devices, a mobile device (e.g., a mobile phone or tablet), and a cloud-based data processing platform. In this proposed system, a WWSD of MEMS motion sensors is used to collect raw data from soccer players. By using BTLE technology, the data is transmitted to the cloud-based data processing platform, which analyzes the data and outputs the results to a mobile device in real-time. A SVM model classification algorithm with an ankle-based attitude angle model is proposed to recognize different motions and assess different skill levels. This intelligent system can be a new paradigm and emerging technology based on wearable sensors, attaining the experience-driven to data-driven transition in the field of sports training and talent selection, and can be easily extended to analyze other foot-related sports motions and skill levels.

In this paper, we propose a system for recognizing soccer motions based on IoT devices, which can recognize users' soccer motions and evaluate the quality of the motions; however, this system still needs to be improved in terms of storage performance and computing speed in the cloud system. The increasing popularity of IoT applications demands the computing power of IoT systems, and edge computing is one of the main methods to enhance the computing speed of IoT applications [32]. In future research, we will try to combine this recognition system with edge computing as well as [33–36], in which authors used edge computing in combination with IoT devices to increase the computational speed of the system and thus reduce its response time.

## Figures and Tables

**Figure 1:** In the IoT system, the motion sensor is attached to the right ankle of the soccer player. The motion data is transmitted via Bluetooth to the Cloud platform for further process.

**Figure 2:** (a) A lithium battery on the back of the board. (b) Circuit board of the WSD. (c) The WSD is attached to the right ankle of a soccer player.

**Figure 3:** The sensor placement and experimental site setting for raw data collection. (a) The WSD is attached to a subject's or player's right ankle. (b) Positions of soccer players to perform passing and shooting.

**Figure 4:** Passing and shooting signal collected from an elite subject. (a) Acceleration of a passing. (b) Angular velocity of a passing. (c) Acceleration of a shooting. (d) Angular velocity of a shooting.

**Figure 5:** The process of soccer motion recognition and assessment system.

**Figure 6:** The elites' and amateurs' passing motion data comparison result: (a), (b), and (c) are the contrast of acceleration on the 3-axes and (d), (e), and (f) are the contrast of angular velocity on 3-axes.

**Figure 7:** Attitude angle: an exploded view of the process of the attitude angle rotation.

**Figure 8:** Comparison of elite's and amateur's attitude angular: (a) is the contrast of pitch, (b) is the contrast of roll, (c) is the contrast of yaw when passing, (d) is the contrast of pitch, (e) is the contrast of roll, and (f) is the contrast of yaw when shooting.

**Figure 9:** With preprocessing, we obtain effective data *S*_*n*−*is*_ for shooting and *S*_*n*−*ip*_ for passing. Add attitude angle for a suitable data form *R*_*n*−*is*_ for shooting and *R*_*n*−*ip*_ for passing. Select key features *F*_*is*_ and *F*_*ip*_ that contribute to maximizing classifier success rates. Combine all samples to obtain *F*_*s*_ and *F*_*p*_.

**Table 1:** Basic and morphology features.

Number	Symbol	Description
1	*R*_*ay*_	Root mean square (RMS) of *y*-axis acceleration
2	*R*_*wx*_	RMS of *x*-axis angular velocity
3	*R*_*wy*_	RMS of *y*-axis angular velocity
4	*R*_*wz*_	RMS of *z*-axis angular velocity
5	*D*_*ax*_	Variance of *x*-axis acceleration
6	*D*_*ay*_	Variance of *y*-axis acceleration
7	*D*_*wy*_	Variance of *y*-axis angular velocity
8	Max_*xy*_	Maximum of *x*-axis acceleration
9	Max_*ay*_	Maximum of *y*-axis acceleration
10	Min_*ay*_	Minimum of *y*-axis acceleration
11	Min_*wz*_	Minimum of *y*-axis angular velocity
12	*S*_*ax*_	Skewness of *x*-axis acceleration
13	*S*_*ay*_	Skewness of *y*-axis acceleration
14	*S*_*az*_	Skewness of *z*-axis acceleration
15	*S*_*wx*_	Skewness of *x*-axis angular velocity
16	*S*_*wy*_	Skewness of *y*-axis angular velocity
17	*S*_*wz*_	Skewness of *z*-axis angular velocity
18	IQR_*ax*_	Interquartile range of *x*-axis acceleration
19	IQR_*ay*_	Interquartile range of *y*-axis acceleration
20	IQR_*az*_	Interquartile range of *z*-axis acceleration
21	IQR_*wx*_	Interquartile range of *x*-axis angular velocity
22	IQR_*wy*_	Interquartile range of *y*-axis angular velocity
23	IQR_*wz*_	Interquartile range of *z*-axis angular velocity
24	Std_*ax*_	Standard deviation of *x*-axis acceleration
25	Std_*wy*_	Standard deviation of *y*-axis angular velocity
26	*M*_*p*_	Mean value of pitch
27	*M*_*r*_	Mean value of roll
28	*M*_*y*_	Mean value of yaw
29	*R*_*p*_	Root mean square of pitch
30	*R*_*r*_	Root mean square of roll
31	*R*_*y*_	Root mean square of yaw
32	Std_*p*_	Standard deviation of pitch
33	Std_*r*_	Standard deviation of raw
34	Std_*y*_	Standard deviation of yaw

**Table 2:** Parameters setting of SVM.

Penalty parameter (*C*)	*γ*	Kernel
1	10^−5^	Linear
500	5× 10^−5^	Polynomial
10^3^	10^−4^	RBF
5× 10^3^	5× 10^−4^	Sigmoid
10^4^	10^−3^	
5× 10^3^	5× 10^−3^	

**Table 3:** Soccer motion recognition accuracies comparison.

Algorithms	Parameter	Accuracy
SVM + angle trajectory model	*C* = 1, *γ* = 10^−4^	0.9
SVM	*C* = 1, *γ* = 5 × 10^−4^	0.88
KNN	*N*_Neighbors = 4	0.85
Decision Tree	Min_Samples Split = 3, max depth = 6	0.86

**Table 4:** The motion recognition result.

Criterion	Motion	Classification	Average
	Passing	Shooting	
Accuracy	0.857	0.885	0.871
Recall	0.96	0.92	0.94
*F*1-score	0.906	0.902	0.904

**Table 5:** Shooting level assessment accuracies comparison.

Algorithms	Parameter	Accuracy
SVM + angle trajectory model	*C* = 1, *γ* = 5 × 10^−5^	0.93
SVM	*C* = 1, *γ* = 10^−4^	0.91
KNN	*N*_Neighbors = 4	0.87
Decision tree	Min_Samples Split = 3, max depth = 6	0.86

**Table 6:** Passing level classification accuracies comparison.

Algorithms	Parameter	Accuracy
SVM + angle trajectory model	*C* = 1, *γ* = 5 × 10^−5^	0.87
SVM	*C* = 1, *γ* = 10^−4^	0.86
KNN	*N*_Neighbors = 4	0.84
Decision Tree	Min_Samples Split = 3, max depth = 6	0.79

**Table 7:** The assessment result for passing and shooting.

Criterion	Skill level of passing		Average	Skill level of shooting		Average
	Elites	Amateurs		Elites	Amateurs	
Accuracy	0.887	0.851	0.869	0.959	0.902	0.931
Recall	0.94	0.8	0.87	0.94	0.92	0.93
*F*1-score	0.913	0.825	0.869	0.949	0.911	0.93

## Data Availability

The soccer motion dataset used to support the findings of this study are currently under embargo while the research findings are commercialized. Requests for data, 12 months after publication of this article, will be considered by the corresponding author.
